The article "Moringa Oleifera aqueous leaf extract down-regulates nuclear factor-kappaB and increases cytotoxic effect of chemotherapy in pancreatic cancer cells" was published in 2013. Journal: BMC Complement Altern Med.

# *Moringa Oleifera* aqueous leaf extract down-regulates nuclear factor-kappaB and increases cytotoxic effect of chemotherapy in pancreatic cancer cells

**DOI:** 10.1186/1472-6882-13-212

**Published:** 2013-08-19

**Authors:** Liron Berkovich, Gideon Earon, Ilan Ron, Adam Rimmon, Akiva Vexler, Shahar Lev-Ari

**Affiliations:** 1 Laboratory of Herbal Medicine and Cancer Research, Tel-Aviv Sourasky Medical Center, Tel-Aviv, Israel

**Keywords:** Moringa Oleifera, Pancreatic cancer, NF-kB, cisplatin

## Abstract

**Background:**

Fewer than 6% patients with adenocarcinoma of the pancreas live up to five years after diagnosis. Chemotherapy is currently the standard treatment, however, these tumors often develop drug resistance over time. Agents for increasing the cytotoxic effects of chemotherapy or reducing the cancer cells’ chemo-resistance to the drugs are required to improve treatment outcome. Nuclear factor kappa B (NF-kB), a pro-inflammatory transcription factor, reportedly plays a significant role in the resistance of pancreatic cancer cells to apoptosis-based chemotherapy. This study investigated the effect of aqueous *Moringa Oleifera* leaf extract on cultured human pancreatic cancer cells - Panc-1, p34, and COLO 357, and whether it can potentiates the effect of cisplatin chemotherapy on these cells.

**Methods:**

The effect of *Moringa Oleifera* leaf extract alone and in combination with cisplatin on the survival of cultured human pancreatic cancer cells was evaluated by XTT-based colorimetric assay. The distribution of Panc-1 cells in the cell cycle following treatment with Moringa leaf extract was evaluated by flow cytometry, and evaluations of protein levels were via immunoblotting. Data of cell survival following combined treatments were analyzed with Calcusyn software.

**Results:**

*Moringa Oleifera* leaf extract inhibited the growth of all pancreatic cell lines tested. This effect was significant in all cells following exposure to ≥0.75 mg/ml of the extract. Exposure of Panc-1 cells to Moringa leaf extract induced an elevation in the sub-G1 cell population of the cell-cycle, and reduced the expression of p65, p-IkBα and IkBα proteins in crude cell extracts. Lastly, *Moringa Oleifera* leaf extract synergistically enhanced the cytotoxic effect of cisplatin on Panc-1 cells.

**Conclusion:**

*Moringa Oleifera* leaf extract inhibits the growth of pancreatic cancer cells, the cells NF-κB signaling pathway, and increases the efficacy of chemotherapy in human pancreatic cancer cells.

## Background

Natural products from plants provide an important source of new drugs and potential pharmaceutical "lead" compounds. Natural products or natural product-derived drugs include 28% of all new chemical entities launched between 1981 and 2002, and 24% of them are semi-synthetic natural product analogues or synthetic compounds based on natural product pharmacophores [1]. Furthermore, many anti-tumor agents in current clinical use are of natural origin, among them taxanes (docetaxel, paclitaxel), Vinca alkaloids (vindesine, vinblastine, vincristine), anthracyclines (idarubicin, daunorubicin, epirubicin), and others. Thus, there is a promising future for the use of natural products derived from plants as anti-tumor agents.

The article "Moringa Oleifera aqueous leaf extract down-regulates nuclear factor-kappaB and increases cytotoxic effect of chemotherapy in pancreatic cancer cells" was published in 2013. Journal: BMC Complement Altern Med.

Adenocarcinoma of the pancreas, the most common form of pancreatic cancer, is the fourth commonest cause of cancer-related mortality worldwide [2]. This cancer is often diagnosed at advanced stages and has a poor prognosis, with fewer than 6% of those patients living as long as five years after diagnosis [2]. The basis of current pancreatic cancer therapy is targeting DNA synthesis using gemcitabine, with or without a second agent like 5-FU or a platinum based agent [3]. Unfortunately, this treatment is limited by a resistance of the cancer cells to these therapies as well as a somatic toxicity [4]. The drug resistance is attributed to several mechanisms: drugs exclusion from the cells, changes in the enzymes metabolizing the drugs, or the cells becoming more resistant to stress and apoptosis [4].

Nuclear factor kappa B (NF-κB) is an essential regulator of the innate and adaptive immunity that, under most conditions, supports proliferation and survival of cells via inhibition of apoptosis [5]. Constitutively active NF-κB signaling that strengthens the malignant cells’ ability to survive has been demonstrated in most tumor cell lines as well as in a variety of patient-derived tumor tissues, including those from pancreatic cancer [6,7]. NF-κB activation has also been directly linked to pancreatic cancer metastatic potential [8]. Although the reason for its constitutive activation in malignant cells has not been fully elucidated, suppression of NF-κB in the majority of these tumors leads to the induction of apoptosis and the subsequent generation of cell death. In addition, several lines of evidence indicate that NF-κB plays a significant role in pancreatic cancer resistance to apoptosis-based chemotherapies, leading to NF-kB being suggested as a potential molecular target for pancreatic cancer therapy [8].

*Moringa Oleifera*, Lam. (Moringaceae) is a tree that grows widely in the tropics and subtropics of Asia and Africa. Its leaves have been traditionally consumed by Asian village people, but it is a relatively novel food material in the western world [9]. *Moringa Oleifera* contains several phytochemicals, some of which are of special interest because of their medicinal properties. Leaves of *Moringa Oleifera* contain flavonoid pigments, such as kaempferol, rhamnetin, isoquercitrin and kaempferitrin. In addition, these leaves are rich in a group of the glycoside compounds, glucosinolates and isothiocyanates [10] as well as beta-sitosterol, glycerol-1-(9-octadecanoate), 3-O-(6'-O-oleoyl-beta-D-glucopyranosyl), beta-sitosterol and beta-sitosterol-3-O-beta-D-glucopyranoside, all of which have demonstrated anti-cancer properties *in-vitro*[11]. An *in-vitro* study using human KB cells as a cancer model has shown that *Moringa Oleifera* leaf extract exerts strong anti-tumor activity [12]. In addition, different leaf extracts of *Moringa Oleifera* generate significant cytotoxic effects on human multiple myeloma cultured cell lines [13].

The article "Moringa Oleifera aqueous leaf extract down-regulates nuclear factor-kappaB and increases cytotoxic effect of chemotherapy in pancreatic cancer cells" was published in 2013. Journal: BMC Complement Altern Med.

The present study examined the effect of *Moringa Oleifera* aqueous leaf extract on the viability and cell cycle of cultured human pancreatic cancer cells, and evaluated its ability to modify the expression of key proteins of the NF-kB signaling pathway. Lastly, this study examined the effect of combined treatments with *Moringa Oleifera* aqueous leaf extract and cisplatin chemotherapy on these cells.

## Methods

### Preparation of *Moringa Oleifera* aqueous extract

Leaves of *Moringa Oleifera* were received from Moringa Arava Ltd, Israel. Moringa Arava grows the *Moringa Oleifera* plant in the Dead Sea area, Israel, where it is grown in rich mineral soil. The plant derived aqueous extract tested in this study was prepared in our laboratory by mixing 1g dried and powdered leaves of *Moringa Oleifera* with 10 mL boiling water for 5 minutes. The mixture was then filtered twice through a 2 μm pore sterile filter paper into a sterile tube. The aqueous extract stock solution (100 mg/mL) was freshly prepared for each set of experiments and stored at 4°C for up to 5 days.

### Cell lines and culture conditions

Human pancreatic cancer cell lines (Panc-1 and COLO-357) were kindly provided by Prof. Ziv Gil (Laboratory for Applied Cancer Research, Tel Aviv Sourasky Medical Center, Israel). Human pancreatic cancer cell line p34 [14], developed from pleural effusion of a pancreatic cancer patient, was kindly provided by Dr. Alex Starr (Laboratory of Lung Biology, Lung and Allergy Institute, Tel Aviv Sourasky Medical Center, Israel). All cells were grown in Dulbecco modified Eagle medium (DMEM) supplemented by 10% heat-inactivated bovine serum, 4.5 g/L glucose, 200 μM L-glutamine, 10 units/ml penicillin and 10 μg/mL streptomycin (Biological Industries, Beit HaEmek, Israel). The cells were incubated at 37°C in a 5% CO_2_ humidified atmosphere. The cells were harvested by trypsin/EDTA solution with 1–2 passages per week in a split ratio of 1:3–5. The 24-hour cell cultures were used in all the experiments.

The article "Moringa Oleifera aqueous leaf extract down-regulates nuclear factor-kappaB and increases cytotoxic effect of chemotherapy in pancreatic cancer cells" was published in 2013. Journal: BMC Complement Altern Med.

### Colorimetric tetrazolium salt (XTT) assay for cell survival

The effect of the treatments tested on the survival of cultured cells was evaluated by XTT-based colorimetric assay (Biological Industries). Typically, 200 μl with 1.5–2x10^3^ cells per well from exponentially growing cultures were plated in 96 micro-well flat-bottom plates. After 24 hours had elapsed, the agents tested were added in calculated concentrations each in three replicate wells and incubated for 72 hours. At the end of the experiment, a freshly prepared mixture of XTT and an activation reagent (PMS) was added into each well (50 μL). Following 2 hours of incubation at 37°C, the optical density (OD) readings were measured at 450 nm using a microplate reader (TECAN Sunrise™ , Switzerland). The measurements were repeated following 3 and 4 hours of incubation, and the time point at which the assay showed optimal OD readings was chosen to calculate the effect of the treatment. When more than one time point fitted these criteria, the results for the different time points were normalized and averaged. Cell survival following treatment was expressed as a percentage of viable cells relative to control value. All the experiments were conducted at least twice, in triplicate wells each, and the results of each experiment were averaged. The preliminary experiments on the selected pancreatic cancer cell lines had demonstrated that the OD readings correlated well (r>0.97–0.99) with the number of seeded cells/well.

### Analysis of synergistic effect of combined treatment

The IC_50_ value of each treatment was calculated on the basis of dose–response curves produced by the XTT assays. In order to determine whether the combined treatment is synergistic or additive, the data on cell survival for each treatment alone and for combined treatment were analyzed with Calcusyn software (Biosoft, Cambridge, UK) that is based on the Chou and Talalay's equations [15]. This software evaluates the combined effect of *Moringa Oleifera* leaf extract and chemotherapeutic agents by calculating the combination index (CI) using the following equation:

$$\mathrm{CI}=\frac{{\left(D\right)}_{1}}{{\left(D_{x}\right)}_{1}}+\frac{{\left(D\right)}_{2}}{{\left(D_{x}\right)}_{2}}$$

Where (D)_1_ and (D)_2_ are the doses of drug 1 and drug 2 in a mixture that inhibits the system x percent and where (Dx)_1_ and (Dx)_2_ are the doses of the drugs that were given individually that inhibited the system x percent. According to the software, CI ≤1 indicates synergism, CI = 1 indicates an additive effect, and CI ≤1 indicates drug antagonism.

The article "Moringa Oleifera aqueous leaf extract down-regulates nuclear factor-kappaB and increases cytotoxic effect of chemotherapy in pancreatic cancer cells" was published in 2013. Journal: BMC Complement Altern Med.

### Immunoblotting analysis

The cells were plated in 10-cm tissue culture dishes for 24 hours at 37°C in a 5% CO_2_ humidified atmosphere. The culture medium was then replaced with a fresh medium supplemented with *Moringa Oleifera* leaf extract for 24 hours. Whole-cell protein samples for immunoblotting were prepared using a proteoJET™ mammalian cell lysis reagent according to standard protocol (Fermentas Life Sciences, Thermo Fisher Scientific). The cytoplasmic and nuclear extracts for immunoblotting were prepared using NucBuster™ protein extraction kit (Novagen® ,U.S.A).

Determination of the protein concentrations was performed using the Bradford assay. Protein from each sample (100 μg) was subjected to electrophoresis in 10% SDS-PAGE and transferred to pure nitrocellulose blotting membranes (Millipore, Bedford, M.A, U.S.A). Membranes were blocked for 1 hour at room temperature with Tris (hydroxymethyl) amino methane saline (TBS) containing 0.05% Tween 20 and 5% non-fat skim milk (BD Bioscience, San Jose, CA). The membranes were then incubated at room temperature in phosphate-buffered solution (PBS) containing 5% milk and the following antibodies (1:200 dilutions): phospho-IκBα (Cell Signaling Technology®, M.A, U.S.A), NF-κB, p65, IκBα and GAPDH (Santa Cruz Biotechnology, Inc., Santa Cruz, CA). Membranes were washed in TBS 0.05% Tween 20, and incubated with either goat, anti-rabbit or rat secondary antibodies (1:1000) conjugated to horseradish peroxidase (Santa Cruz Biotechnology, Inc. U.S.A). Detection was by SuperSignal® West Pico from Pierce BioLynx Inc. (Brockville, Ontario, Canada) reagent.

### Flow cytometry (FACS) analysis of cell cycle

The distribution of Panc-1 cells (intact and treated with *Moringa Oleifera* leaf extract for 24 hours) in the cell cycle was evaluated by flow cytometry. FACS analysis was used to detect sub-diploid apoptotic cells, and trypan blue assay was used to discriminate between necrotic and apoptotic cells. The cells (0.5-1.0x10^6^ cells/plate) were collected following treatment, washed with cold PBS, fixed in ice cold 70% ethanol and kept at −20°C for 24–48 hours. The pellets were washed in cold PBS and suspended in PBS containing 0.1% Triton-X and 30 mg/mL DNAse-free RNAse A (Sigma-Aldrich, Israel) for 6 hours at room temperature. Approximately one minute before the cells were analyzed, propidium iodide (Sigma) in PBS was added at a final concentration of 10 μg/mL. The samples were analyzed using a FACSCallibur instrument (BD Bioscience). Data were processed with BD Bioscience software.

### Statistical analysis

The results for each variant of treatment in these experiments were represented as an average of 2–4 experiments, and each arm was performed in triplicate. The mean values and standard errors were calculated for each time point from the pooled normalized data. The statistical significance of the difference between groups was determined by the two-tailed Student’s *t*-test. Values of *p* < 0.05 were considered significant.

The article "Moringa Oleifera aqueous leaf extract down-regulates nuclear factor-kappaB and increases cytotoxic effect of chemotherapy in pancreatic cancer cells" was published in 2013. Journal: BMC Complement Altern Med.

## Results

The antiproliferative and apoptotic effects of the aqueous leaf extract of *Moringa oleifera* have been previously evaluated in KB cultured human tumor cells [12], where the extract was used in up to 200 μg/mL final concentration. Thus, for our survival experiments of cultured pancreatic cancer cells we started looking for an effect around 0.1 mg/mL and upraised it according to our results.

### Effect of *Moringa Oleifera* leaf extract on survival and cell cycle of pancreatic cancer cells

The effect of *Moringa Oleifera* leaf extract (0.1-2.0 mg/mL) on the survival of cultured pancreatic cancer cells was evaluated following exposure for 72 hours. As shown in Figure 1, *Moringa* extract inhibited the growth of all three tested cell lines. Panc-1 cells were more susceptible to the treatment (IC_50_ = 1.1 mg/ml) compared to COLO 357 (IC_50_ =1.8 mg/ml) and p34 cells (IC_50_ = 1.5 mg/ml). There was a significant inhibition of Panc-1 cell survival at an extract concentration of 0.75 mg/mL. There was also a significant inhibitory effect at a higher concentration (1.5 mg/mL) in the two other cell lines. Moreover, treatment with 2 mg/mL *Moringa* extract resulted in a 98% reduction of Panc-1 cell survival.

**Figure 1:** **Effect of *Moringa Oleifera *leaf extract on the viability of Panc-1, COLO 357 and p34 pancreatic cancer cells.** The cells were plated in 96-well plates and treated in triplicates with *Moringa Oleifera* leaf extract for 3 days. Cell survival was assessed using XTT-based cell proliferation assay, and is indicated after normalization to the control group. The significance of the effect is indicated as *p ≤ 0.05 and **p ≤ 0.001.

We also evaluated the distribution of Panc-1 cells in the cell cycle following 24 hours exposure to *Moringa Oleifera* leaf extract using flow cytometry analysis of propidium iodide-stained cells. It revealed a dose-dependent significant increase of the percentage of cells in the sub-G1 phase, characterized by a very low DNA content, following *Moringa* extract treatment (Figure 2A&B). This indicated a fragmentation of the DNA as a result of progressive cell apoptosis. Importantly, *Moringa* extract treatment also induced significant (*p* < 0.05) apoptosis in Panc-1 cancer cells at the minimal evaluated concentration of 0.25 mg/mL. The induction of apoptosis was especially high (up to 30%) at a concentration of 0.75 mg/mL.

The article "Moringa Oleifera aqueous leaf extract down-regulates nuclear factor-kappaB and increases cytotoxic effect of chemotherapy in pancreatic cancer cells" was published in 2013. Journal: BMC Complement Altern Med.

**Figure 2:** **Effect of *Moringa Oleifera *leaf extract on the distribution of Panc-1 cells in the cell cycle.** (**A**) Representative histograms of cell distribution following *Moringa Oleifera* leaf extract treatments. (**B**) Data summarized from three independent experiments (%). The cells were treated with the extract for 24 hours, collected, washed and fixed in 70% ice-cold ethanol. Prior to the analysis, the cells were suspended in 0.1% Triton-X with 30 mg/ml DNAse-free RNAse A for 6 hrs. Propidium iodide was added several minutes before cell analysis by flow cytometry. The significance of the effect, relatively to non-treated cells (control), is indicated as *p ≤ 0.05 and **p ≤ 0.001.

### Effect of *Moringa Oleifera* leaf extract on NF-κB signaling pathway in pancreatic cancer cells

*Moringa Oleifera* leaf extract treatment of Panc-1 cells down-regulated the expression of key NF-κB signaling pathway proteins (Figure 3). The treatment of the cells with 0.25 mg/mL extract for 24 hours resulted in a down-regulation of p65, phospho-IκBα and IκBα proteins levels compared to untreated cells (Figure 3A). Treatments with 0.75 and 1.5 mg/mL *Moringa* extract reduced or eliminated more significantly the presence of all three proteins of the NF-κB signaling pathway. Moreover, p65 protein subunit levels have decreased in Panc-1 cells nuclei as a result of treatments with 0.1 - 1.5 mg/mL *Moringa* extract. These data suggest that *Moringa* extract attenuated pancreatic cancer cell’s survival ability, at least in part, by targeting the NF-κB signaling pathway.

**Figure 3:** **Effect of *Moringa Oleifera *leaf extract on the expression of p65 NF-kB, IkB and p-IkB proteins in Panc-1. (A)** Protein expressions in crude lysates of the cells treated with *Moringa Oleifera* leaf extract (0–1.5 mg/mL) for 24 hours. **(B)** Expression of p65 in nuclear extracts of the cells treated with *Moringa Oleifera* leaf extract. Protein expression was analyzed by Western blot. GAPDH and ß-actin were used to demonstrate the quantity of standard proteins in the samples tested.

### Combined effect of *Moringa Oleifera* leaf extract and cisplatin

Based on the ability of *Moringa* extract to inhibit the NF-κB signaling pathway, we hypothesized that its extract treatment would sensitize pancreatic cancer cells to chemotherapy. We therefore tested the cytotoxic effect of several combinations of *Moringa Oleifera* leaf extract with cisplatin on Panc-1 cells. Since a synergistic effect was expected, both the agents were used in the concentrations of a low inhibitory effect on proliferation of Panc-1 cells. As shown in Figure 4, all the tested combinations demonstrated an inhibitory effect higher than the effects of each agent alone. The analysis of these data by Calcusyn software, presented in Figure 4 and summarized in the Table 1, clearly demonstrated that the combined *Moringa Oleifera* leaf extract and cisplatin regimen resulted in strong synergistic (CI = 0.1–0.3) or synergistic (CI = 0.3–0.7) effects.

The article "Moringa Oleifera aqueous leaf extract down-regulates nuclear factor-kappaB and increases cytotoxic effect of chemotherapy in pancreatic cancer cells" was published in 2013. Journal: BMC Complement Altern Med.

**Figure 4:** **Combined treatments effect of *Moringa Oleifera *leaf extract with cisplatin on the viability of Panc-1 cells. (A)** Cell viability following treatments of *Moringa Oleifera* leaf extract, cisplatin and combined treatments of increasing concentrations of the extract and cisplatin for 3 days. **(B)** Normalized isobologram of *Moringa Oleifera* leaf extract with cisplatin treatments shown in compound A. **(C)** Median-effect plot curve of *Moringa Oleifera* leaf extract, cisplatin and *Moringa Oleifera* leaf extract with cisplatin shown in compound A. The cells were treated with each agent alone or in combination for 3 days. Cell viability was evaluated using XTT-based cell proliferation assay. Data was analyzed by Calcusyn software.

**Table 1:** **Calculated Combination Index (CI) of the effect of combined treatments with *Moringa Oleifera *leaf extract and cisplatin on Panc-1 cells viability**

**Combination index (CI)**	**Cisplatin (μM)**	**Moringa (mg/mL)**
**0.348**	**0.3**	**0.25**
**0.517**	**0.3**	**0.50**
**0.652**	**0.3**	**0.75**
**0.218**	**1.0**	**0.25**
**0.379**	**1.0**	**0.50**
**0.539**	**1.0**	**0.75**
**0.156**	**3.0**	**0.25**
**0.375**	**3.0**	**0.50**
**0.504**	**3.0**	**0.75**

The cells were treated as described in Figure 4. Cell viability was evaluated using XTT-based cell proliferation assay. Data was analyzed using Calcusyn software.

## Discussion

The results of this study show that *Moringa Oleifera* leaf extract can significantly inhibit the growth of cultured human pancreatic carcinoma cells as well as its cell-cycle progression, in a concentration-dependent manner. Notably, the reduction of Panc-1 cells viability reached 100% following exposure to 2 mg/mL of *Moringa* extract (Figure 1). To the best of our knowledge, this is the first time that *Moringa Oleifera* was shown to have an effect on pancreatic carcinoma cells. The exposure of Panc-1 cells to *Moringa Oleifera* leaf extract also reduced the overall expression of key NF-κB family proteins in the cells, as well as the levels of p65 protein subunit in the cell nuclei (Figure 3). Consequently, this extract could inhibit the NF-κB signaling cascade execution of target gene transcription. Active NF-κB signaling was shown to strengthen the pancreatic cancer cell’s ability to survive, and that suppression of NF-κB leads to induction of apoptosis and thus generation of cell death [8]. Inhibition of the NF-κB signaling cascade by Moringa extract explains, at least in part, its attenuating effect on the survival of pancreatic cancer cells, as observed on the viability assay (Figure 1).

The article "Moringa Oleifera aqueous leaf extract down-regulates nuclear factor-kappaB and increases cytotoxic effect of chemotherapy in pancreatic cancer cells" was published in 2013. Journal: BMC Complement Altern Med.

Several lines of evidence indicate that NF-κB plays a significant role in the resistance of pancreatic cancer to apoptosis-based chemotherapies. Therefore, the NF-κB signaling pathway was suggested as a potential molecular target for combined therapy of pancreatic cancer [8,16]. Cisplatin is a platinum-based chemotherapeutic agent that is known to have a minimal clinical efficacy in pancreatic cancer due to tumor chemoresistance mechanisms [4]. It has been shown in other human cancer models that increased efficacy of cisplatin may be achieved by NF-κB inhibitors in cancer cells [17,18]. Therefore, we hypothesized that the effect of *Moringa Oleifera* leaf extract on the inhibition of the NF-κB pathway may increase the efficacy of cisplatin. As shown in Figure 4 and summarized in Table 1, combined therapy of *Moringa Oleifera* leaf extract with cisplatin demonstrated strong (CI = 0.1–0.3) or moderate (CI = 0.3–0.7) synergistic effects in Panc-1 cells, respectively. This indicates that the treatment of pancreatic cancer with cisplatin in combination with *Moringa Oleifera* leaf extract may be a clinical therapeutic option for this chemoresistant cancer.

The past decade has witnessed the establishment of herbal medicine as a rich source of new "western medicine" drugs for multiple conditions, including cancer. These herbs are often traditionally consumed by particular populations, presenting an advantage in terms of laying rest to toxicity concerns. Herbs and their bioactive metabolites have been reported to be anti-neoplastic both in experimental and clinical studies [19,20]. *Moringa Oleifera* leaves contain flavonoid pigments, such as kaempferol, rhamnetin, isoquercitrin and kaempferitrin. Flavonoid compounds have various biological activities, including anti-inflammatory and anti-cancer ones [21], and may be mediating, at least in part, the effects shown here. In addition, the *Moringa Oleifera* leaves are rich in a group of the glycoside compounds, glucosinolates and isothiocyanates [10], as well as in beta-sitosterol, glycerol-1-(9-octadecanoate), 3-O-(6'-O-oleoyl-beta-D-glucopyranosyl), beta-sitosterol and beta-sitosterol-3-O-beta-D-glucopyranoside, all of which have demonstrated anti-cancer properties *in-vitro*[11] and may have also contributed to the effects we exhibit. Since this work does not include the isolation of bioactive compounds from the *Moringa Oleifera* leaf extract, we are not able to propose one or more specific active compounds to be mediating the cellular anti-cancer effects demonstrated in our results. Moreover, it is possible that our findings can be attributed to additive or synergistic effects of several bioactive compounds from the extract and not to a single one. Further research on anti-cancer effects of specific bioactive metabolites derived from Moringa Oleifere is warranted.

The article "Moringa Oleifera aqueous leaf extract down-regulates nuclear factor-kappaB and increases cytotoxic effect of chemotherapy in pancreatic cancer cells" was published in 2013. Journal: BMC Complement Altern Med.

Toxicity has been a limiting factor in clinical pancreatic cancer treatment: combined therapy with cisplatin and gemcitabine has shown promising results in phase II and III trials, but it was followed by severe toxicity and therefore has not been approved as a standard of care [4]. This should not be the case regarding *Moringa Oleifera Lam*, since an acute toxicity test carried out using male Wistar albino mice, estimated the LD(50) of orally administered aqueous leaf extract of *Moringa oleifera Lam.* to be around 1585 mg/kg for a single administration [22]. The aqueous leaf extract of *Moringa oleifera* is, therefore, considered relatively safe when administered orally and its acquisition of permission for clinical use highly probable.

Still, future studies need to be conducted to evaluate and quantify the therapeutic index of *Moringa Oleifera* leaf extract applicable to pancreatic cancer patients in the clinical setting.

## Conclusions

*Moringa Oleifera* leaf extract inhibits the NF-κB signaling pathway and increases the efficacy of chemotherapy in human pancreatic cancer cells.

## Abbreviations

NF-κB: Nuclear factor kappa-B; XTT: 2,3-bis-(2-methoxy-4-nitro-5-sulfophenyl)-2H-tetrazolium-5-carboxanilide; CI: Combination Index; PBS: Phosphate-buffered solution; GAPDH: Glyceraldehyde 3-phosphate dehydrogenase; OD: Optical density.

## Competing interest

The authors declare that they have no competing interests.

## Authors’ contributions

LB planned the study’s experiments, conducted the cell culture experiments, analyzed the signaling assays and prepared the manuscript. SLA, AR and AV performed the statistical analysis and data calculations. GE and IR assisted with the manuscript. SLA conceived the study and gave final approval of the manuscript. All authors read and approved the final manuscript.

## Pre-publication history

The pre-publication history for this paper can be accessed here:

http://www.biomedcentral.com/1472-6882/13/212/prepub
